# A Clinical Study on the Effect of Different Ratios of Recombinant Human Bone Morphogenetic Protein-2 Compound to Autogenous Bone on Cervical Interbody Fusion Based on Smart Healthcare

**DOI:** 10.1155/2021/1033900

**Published:** 2021-12-16

**Authors:** Xinzhu Zhang, Kun Zhao, Feng Yuan, Youlai Yu, Bin Deng

**Affiliations:** ^1^Department of Spinal Surgery, Affiliated Hospital of Xuzhou Medical University, Xuzhou, Jiangsu 221000, China; ^2^Clinical Laboratory, Xuzhou Maternal and Child Health Care Hospital, Xuzhou, Jiangsu 221000, China

## Abstract

With an increasing elderly population worldwide, the incidence of spine degenerative diseases with neck and shoulder pain as the main symptom is rising obviously, which has now become one of the important and difficult problems in sociomedical science. This study was to explore the effects of different ratios of recombinant human bone morphogenetic protein-2 (rhBMP-2) compound to the autogenous bone on cervical interbody fusion. 90 cervical degeneration patients with the need of surgical treatment admitted to our hospital from January 2019 to January 2020 were selected as the research objects and equally divided into group A, group B, and group C according to the order of admission, with 30 cases in each group and the ratios of rhBMP-2 compound to autogenous bone being 2 : 1, 1 : 1, and 1 : 2 respectively, and standard anterior cervical diskectomy and fusion (ACDF) treatment was performed to all patients to compare their surgery-related indexes, the Japanese Orthopaedic Association (JOA) score, the visual analog scale (VAS) score, the effect of cervical interbody fusion, and the postoperative complication rate (CR). Compared with group A and group C, group B achieved the significantly better surgery-related indexes (*P* < 0.05), significantly higher postoperative JOA scores (*P* < 0.05), significantly lower postoperative neck and upper limb VAS scores (*P* < 0.05), significantly better effect of cervical interbody fusion (*P* < 0.05), and significantly lower postoperative CR (*P* < 0.05). 1 : 1 is the best ratio of rhBMP-2 compound to the autogenous bone, for it can optimize patients' perioperative indexes, reduce the postoperative pain, lower the possibility of complications, and improve the effect of cervical interbody fusion, which should be promoted and applied in practice.

## 1. Introduction

With an increasing elderly population worldwide, the incidence of spine degenerative diseases with neck and shoulder pain as the main symptom is rising obviously, which has now become one of the important and difficult problems in sociomedical science [1–3]. The anterior cervical diskectomy and fusion (ACDF) is an important procedure for treating cervical diseases. Generally, patients can achieve relatively desirable outcomes after ACDF, but several studies in recent years have reported that many factors affect the prognosis of such patients, and if the surgical segments cannot achieve effective fusion, problems such as loosening of internal fixation will occur and then seriously affect the postoperative recovery. Therefore, selecting the appropriate fusion material is the key to improving the rate of cervical interbody fusion for ACDF [4–6]. At present, the fusion materials commonly used in practice are mainly the autogenous or alloplastic bone, in which the autogenous bone is limited in extraction and the alloplastic bone may elevate the possibility of ACDF failure, so both of them do not have good application conditions. Nowadays, the development of substitute materials such as the artificial bone has enabled ACDF with more material choices. Scholars have found that the recombinant human bone morphogenetic protein-2 (rhBMP-2) can accelerate the generation rate of cells, enhance the defect repairability of bone, and then fully optimize the effect of cervical interbody fusion [7–10]. It is an indisputable fact in academia that rhBMP-2 can improve the fusion rate of ACDF, but the optimal dosage is still not clear. Based on this, to explore the effect of different ratios of rhBMP-2 compound to the autogenous bone on cervical interbody fusion, 90 cervical degeneration patients with the need of surgical treatment admitted to our hospital from January 2019 to January 2020 were selected for the study, and the summary results are as follows.

## 2. Materials and Methods

### 2.1. General Information

90 cervical degeneration patients with the need of surgical treatment admitted to our hospital from January 2019 to January 2020 were selected as the research objects and equally divided into group A, group B, and group C according to the order of admission, with 30 cases in each group, the ratios of the rhBMP-2 compound to the autogenous bone being 2 : 1, 1 : 1, and 1 : 2 respectively, and no statistical difference between the patients' general information (*P* > 0.05), as given in Table 1. This study was approved by the hospital ethics committee.

### 2.2. Inclusion Criteria

The inclusion criteria for the study were as follows. (1) Patients or their family members fully understood the study process and signed the informed consent; (2) patients had nerve root or spinal spondylosis symptoms and needed cervical fusion surgery; and (3) patients were diagnosed with single-segment degenerative cervical spondylotic myelopathy or spinal cord cervical disc herniation [11].

### 2.3. Exclusion Criteria

The exclusion criteria for the patients in the study were as follows. (1) Presence of mental problems or inability to communicate with others; (2) presence of ossification of the posterior longitudinal ligament; (3) prior treatment of cervical vertebra surgery; (4) presence of other organic diseases; and (5) failure to cooperative with the study for other reasons.

### 2.4. Methods

#### 2.4.1. Surgical Methods

(1) Standard ACDF treatment was performed on all patients by surgeons of the same group. (2) Half an hour before the surgery, patients were infused with antibiotics to prevent intraoperative infection and were lying on their back under general anesthesia. (3) Patients' neck was remained straightened, and the incision was made at the right front part of the neck, the surgical space was located with the C-arm X-ray apparatus (BV Pulsera, NMPA (I) 20083303102); before the separation between the arterial sheath and the tracheoesophageal sheath reached in front of the vertebral body, the bone material at the front margin of the upper vertebrae was taken out, and all the removed osteophytes were reserved. (4) Patients' intervertebral spaces were spread with a spreader (Changzhou Kanghui Medical Innovation Co., Ltd., Jiangsu Changzhou MPA Certified No. (2008) 1100111), the anterior intervertebral disc was excised with a long-pointed knife, and then, the disc and the posterior border of the vertebral bone cone were removed with the curette. (5) When the scope of decompression on both sides reached the Luschka joint and that on the posterior aspect reached the posterior longitudinal ligament or dura mater, the intervertebral foramen was enlarged, and the nerve root was thoroughly decompressed. (6) The superior and inferior vertebral cartilaginous laminae were curetted, leaving the intact cortical bone beneath the lamina to prevent collapse of the intervertebral space. (7) The cages of each group were filled with the established ratio of bone graft (containing rhBMP-2, Hangzhou Huadong Medicine Investment Co., Ltd.) and bone granules and then implanted into the intervertebral space to maintain the fine indirect contact with the adjacent vertebral endplate. (8) The surgical segments were fixed intraplate, the incision was rinsed thoroughly, 1 negative pressure drainage tube was indwelt in place, and the suture was performed finally.

#### 2.4.2. Postoperative Treatment

(1) The patients were given antibiotics once to prevent infection within 24 h after surgery, while dexamethasone (Guangdong Huanan Pharmaceutical Group Co., Ltd., NMPA Approval No. H44024469) and dehydration drugs were applied to relieve the postoperative edema. (2) The drainage tube was removed when the drainage volume was below 30 ml in 1-2 days after surgery, patients could wear the cervical collar and move around 1 day later, and all cervical fore and anterolateral X-ray films were reviewed after drainage tube removal. (3) Patients had their incision sutures removed 6 days after surgery and wore the cervical collar for protection for 6 weeks.

### 2.5. Observation Criteria

1. Surgery-related indexes, which included the surgery time, intraoperative blood loss, postoperative drainage volume, and hospitalization time
2. JOA score: a total of 17 scoring items were included, of which 4 points each for the motor function of four limbs, 2 points each for the sensory function of the body and four limbs, and 3 points for the bladder function. Scores of 0–4 regarded as patients with severe condition had most or completely paralyzed limbs and were unable to take care of themselves; scores of 5–8 regarded as patients with serious condition had partially functional limbs but lost the ability to work; scores of 9–12 regarded as patients with moderate condition had limbs with movement disorders and could do some simple works; and scores of 13–16 regarded as patients with mild condition had slight movement disorders and were essentially able to live and work normally [12, 13]. The JOA score was investigated at 1 month (*T*_1_), 2 months (*T*_2_), 3 months (*T*_3_), and 6 months (*T*_4_) after surgery.
3. VAS score: it was used to evaluate patients' pain and numbness in the neck and upper limbs, with higher scores indicating stronger pain [14]. The VAS score was investigated at 1 month (*T*_1_), 2 months (*T*_2_), 3 months (*T*_3_), and 6 months (*T*_4_) after surgery.
4. Effect of cervical interbody fusion: it was considered as a fine effect if the imaging examination showed that the trabecular bone crossed the fusion gap or the vertebral anterior and posterior margins, the bone bridges were formed, the fusion gap was free of displacement and collapse, and the fusion site had no radiolucent line and no osteonecrosis. The effect of cervical interbody fusion was investigated at 3 months (*T*_3_) and 6 months (*T*_4_) after surgery.
5. Postoperative complication rate (CR): neck complications included anterior cervical edema, dysphagia, and cerebrospinal leakage; donor site complications included infection and fracture of anterior superior iliac spine; and internal fixation-related complications included titanium plate screw fracture and screw loosening. The number of patients who developed complications was counted, and the proportion was calculated.

### 2.6. Statistical Processing

In this study, the data processing software was SPSS 18.0, the picture drawing software was GraphPad Prism 7 (GraphPad Software, San Diego, USA), items included were enumeration data and measurement data, methods used were the *X*^2^ test and *t* test, and differences were considered statistically significant at *P* < 0.05.

## 3. Results

### 3.1. Comparison of Patients' Surgery-Related Indexes

Patients' surgery-related indexes of group B were significantly better than those of group A and group C (*P* < 0.05), with statistically significant differences, as given in Table 2.

### 3.2. Comparison of Patients' JOA Scores

Patients' JOA scores of group B were significantly higher than those of group A and group C (*P* < 0.05), with statistically significant differences, as shown in Figure 1.

### 3.3. Comparison of Patients' VAS Scores

Patients' postoperative neck and upper limb VAS scores of group B were significantly lower than those of group A and group C (*P* < 0.05), with statistically significant differences, as shown in Figures 2 and 3.

### 3.4. Comparison of the Effect of Cervical Interbody Fusion

The effect of cervical interbody fusion of group B was significantly better than that of group A and group C (*P* < 0.05), with statistically significant differences, as given in Table 3.

### 3.5. Comparison of Patients' Postoperative CR

The postoperative CR of group B was significantly lower than that of group A and group C (*P* < 0.05), with statistically significant differences, as given in Table 4.

## 4. Discussion

ACDF is an important way of treating cervical diseases, and the selection of fusion materials plays a decisive role in patient outcomes. Both autogenous and allogeneic bone materials commonly used in the clinic are limited in application, while the novel rhBMP-2, which helps the mesenchymal cells differentiate to form osteocytes, promotes the transformation of the artificial synthetic bone into bone tissue, enhances the cervical fusion rate, and shows good surgical effects of ACDF [8, 15–17]. Recently, it has been documented that rhBMP-2 can lead to severe complications such as inflammatory response and wound infection, and high-dose rhBMP-2 may even cause cancer [18]; therefore, strengthening the research on the dosage of rhBMP-2 is essential. In this study, the results showed that patients' postoperative CR of group B was significantly lower than that of group A and group C (*P* < 0.05), indicating that the highest fusion rate was achieved when the ratio of rhBMP-2 compound to the autogenous bone was 1 : 1, because under such ratio, the biomechanical advantages of the two materials could be sufficiently combined to reduce the complications caused by the dosage of rhBMP-2 and fully enhance the safety and feasibility of rhBMP-2 therapy. In addition, the dosage of rhBMP-2 selected for group A was higher, but its CR was not significantly higher than that of group C, which may be related to the rhBMP-2 carrier used. A good rhBMP-2 carrier can accelerate the migration of bone cells, produce nontoxic degradation products, control the overall CR at a low level, and protect patients' body health.

Patients' surgery-related indexes of group B were significantly better than those of groups A and C (*P* < 0.05), which was consistent with the findings of scholars Ramly E P et al. Their research showed that the application of rhBMP-2 compound as a bone grafting material could effectively shorten the surgery time of ACDF and reduce the intraoperative blood loss and postoperative drainage volume of patients; moreover, a reasonable dose would further optimize patients' perioperative indexes and accelerate the rehabilitation progress [19].

Patients' postoperative JOA scores of group B were significantly higher than those of groups A and C (*P* < 0.05), indicating that the ratio of bone graft materials of 1 : 1 could exert a more desirable fusion effect. rhBMP-2 can not only relieve the spinal cord compression but also accelerate the differentiation rate of monocytes, promote chondrogenesis, and then induce new bone formation [20–22], explaining the fact that the effect of cervical interbody fusion of patients in group B was significantly better than that of groups A and C (*P* < 0.05). Therefore, a reasonable ratio of rhBMP-2 can increase the fine rate of interbody fusion and improve the wound healing progress comprehensively at 3 months after surgery.

## 5. Conclusion

In the scholar Ishida W's study, the neck and upper limb VAS scores at 3 months after surgery of patients given 1 mg rhBMP-2 were (2.81 ± 1.20) and (2.44 ± 0.78), respectively, which were significantly lower than those of patients given 2 mg rhBMP-2 and patients treated with completely autogenous bone grafting (*P* < 0.001) [22], indicating that rhBMP-2 could relieve patients' postoperative pain. In this study, the postoperative neck and upper limb VAS scores of patients in group B were significantly lower than those in groups A and C (*P* < 0.05), which was similar to Ishida W's study results. Patients in group B recovered faster, had lower CR, and were less affected by adverse symptoms after surgery; therefore, they suffered from less pain.

In conclusion, the best ratio of rhBMP-2 compound to the autogenous bone is 1 : 1, for it can optimize patients' perioperative indexes, reduce the postoperative pain, lower the possibility of complications, and improve the effect of cervical interbody fusion, which should be promoted and applied in practice.

## Figures and Tables

**Figure 1:** Comparison of patients' JOA scores ($\bar{X}\pm s$, points). The horizontal axis from left to right shows the time points of 1 month (*T*_1_), 2 months (*T*_2_), 3 months (*T*_3_), and 6 months (*T*_4_) after surgery, and the vertical axis shows the JOA score (points); the black area shows group A, the dark gray area shows group B, and the light gray area shows group C. The JOA scores at *T*_1_ of group A, group B, and group C were (10.89 ± 0.56), (11.31 ± 0.74), and (10.56 ± 0.57), respectively; the JOA scores at *T*_2_ of group A, group B, and group C were (11.74 ± 0.54), (13.11 ± 1.23), and (11.56 ± 0.57), respectively; the JOA scores at *T*_3_ of group A, group B, and group C were (12.14 ± 0.54), (14.56 ± 1.10), and (12.23 ± 0.45), respectively; and the JOA scores at *T*_4_ of group A, group B, and group C were (13.41 ± 0.78), (14.89 ± 1.21), and (13.26 ± 0.89), respectively. ^*∗*^*P* < 0.05.

**Figure 2:** Comparison of patients' upper limb VAS scores ($\bar{X}\pm s$, points). The horizontal axis from left to right shows the time points of 1 month (*T*_1_), 2 months (*T*_2_), 3 months (*T*_3_), and 6 months (*T*_4_) after surgery, and the vertical axis shows the VAS score (points); the dot line shows group A, the block line shows group B, and the triangle line shows group C. The VAS scores at *T*_1_ of group A, group B, and group C were (3.11 ± 1.21), (2.21 ± 1.24), and (3.05 ± 1.20), respectively; the VAS scores at *T*_2_ of group A, group B, and group C were (3.02 ± 0.78), (2.10 ± 0.85), and (2.99 ± 0.86), respectively; the VAS scores at *T*_3_ of group A, group B, and group C were (2.45 ± 0.96), (1.41 ± 0.85), and (2.36 ± 0.74), respectively; and the VAS scores at *T*_4_ of group A, group B, and group C were (1.99 ± 0.68), (1.01 ± 0.69), and (1.87 ± 0.67), respectively ^*∗*^*P* < 0.05.

**Figure 3:** Comparison of patients' neck VAS scores ($\bar{X}\pm s$, points). The horizontal axis from left to right shows the time points of 1 month (*T*_1_), 2 months (*T*_2_), 3 months (*T*_3_), and 6 months (*T*_4_) after surgery, and the vertical axis shows the VAS score (points); the dot line shows group A, the block line shows group B, and the triangle line shows group C. The VAS scores at *T*_1_ of group A, group B, and group C were (3.89 ± 1.20), (3.10 ± 1.15), and (3.91 ± 1.26), respectively; the VAS scores at *T*_2_ of group A, group B, and group C were (3.56 ± 1.11), (2.68 ± 1.52), and (3.52 ± 1.10), respectively; the VAS scores at *T*_3_ of group A, group B, and group C were (2.89 ± 1.23), (2.29 ± 1.02), and (2.86 ± 1.11), respectively; and the VAS scores at *T*_4_ of group A, group B, and group C were (2.55 ± 1.20), (1.91 ± 1.00), and (2.52 ± 1.23), respectively. ^*∗*^*P* < 0.05.

**Table 1:** Comparison of patients' general information.

Group	*N*	Age (years old)	Weight (kg)	Diagnostic classification (cases) Nerve Root spinal	
Group A	30	54.89 ± 5.26	62.12 ± 6.21	29	31
Group B	30	55.01 ± 5.24	62.14 ± 6.23	30	30
Group C	30	54.99 ± 5.32	62.10 ± 6.25	28	32

**Table 2:** Comparison of patients' surgery-related indexes ($\bar{X}\pm s$).

Group	*N*	Surgery time (min)	Intraoperative blood loss (ml)	Postoperative drainage volume (ml)	Hospitalization time (d)
Group A	30	99.15 ± 26.48	140.57 ± 32.46	89.12 ± 20.56	9.45 ± 5.11
Group B	30	85.56 ± 25.24^*∗∗∗*^	117.56 ± 35.89^*∗*^^*∗∗*^	71.56 ± 21.12^*∗∗∗*^	6.98 ± 4.26^*∗∗∗*^
Group C	30	98.58 ± 24.26	146.89 ± 15.26	90.12 ± 21.15	9.41 ± 4.95

^*∗*^Comparison with group A, *P* < 0.05. ^*∗∗*^Comparison with group C, *P* < 0.05.

**Table 3:** Comparison of the effect of cervical interbody fusion (*n* (%)).

Group	*N*	Fine fusion rate at 3 months after surgery	Fine fusion rate at 6 months after surgery
Group A	30	24 (80.0)	26 (86.7)
Group B	30	29 (96.7)^*∗*^^*∗∗*^	30 (100.0)^*∗*^^*∗∗*^
Group C	30	24 (80.0)	25 (83.3)

^*∗*^Comparison with group A, *P* < 0.05. ^*∗∗*^Comparison with group C, *P* < 0.05.

**Table 4:** Comparison of patients' postoperative CR (*n* (%)).

Group	Group A	Group B	Group C
Neck complications			
Anterior cervical edema	0 (0.0)	0 (0.0)	0 (0.0)
Dysphagia	3 (10.0)	1 (3.3)	3 (10.0)
Cerebrospinal leakage	1 (3.3)	0 (0.0)	2 (6.7)

Donor site complications			
Infection	2 (6.7)	0 (0.0)	1 (3.3)
Fracture of anterior superior iliac spine	2 (6.7)	1 (3.3)	1 (3.3)

Internal fixation-related complications			
Titanium plate screw fracture	0 (0.0)	0 (0.0)	1 (3.3)
Screw loosening	1 (3.3)	0 (0.0)	0 (0.0)
Total times of complication	9 (30.0)	2 (6.7)^*∗*^^*∗∗*^	8 (26.7)

^*∗*^Comparison with group A, *P* < 0.05. ^*∗∗*^Comparison with group C, *P* < 0.05.

## Data Availability

The datasets used and/or analyzed during the current study are available from the corresponding author upon request.
